# Augmentation-Consistent Clustering Network for Diabetic Retinopathy Grading with Fewer Annotations

**DOI:** 10.1155/2022/4246239

**Published:** 2022-03-28

**Authors:** Guanghua Zhang, Keran Li, Zhixian Chen, Li Sun, Jianwei zhang, Xueping Pan

**Affiliations:** ^1^Department of Intelligence and Automation, Taiyuan University, Taiyuan 030000, China; ^2^The Affiliated Eye Hospital of Nanjing Medical University, Nanjing, China; ^3^Affiliated Hospital of Integrated Traditional Chinese and Western Medicine, Nanjing University of Chinese Medicine, Nanjing 210028, China; ^4^Jiangsu Provincial Academy of Traditional Chinese Medicine, Nanjing 210028, China; ^5^Technical Aspects of Multimodal Systems (TAMS), University of Hamburg, Hamburg 22527, Germany; ^6^The First People's Hospital of Huzhou, Huzhou 313000, China

## Abstract

Diabetic retinopathy (DR) is currently one of the severe complications leading to blindness, and computer-aided, diagnosis technology-assisted DR grading has become a popular research trend especially for the development of deep learning methods. However, most deep learning-based DR grading models require a large number of annotations to provide data guidance, and it is laborious for experts to find subtle lesion areas from fundus images, making accurate annotation more expensive than other vision tasks. In contrast, large-scale unlabeled data are easily accessible, becoming a potential solution to reduce the annotating workload in DR grading. Thus, this paper explores the internal correlations from unknown fundus images assisted by limited labeled fundus images to solve the semisupervised DR grading problem and proposes an augmentation-consistent clustering network (ACCN) to address the above-mentioned challenges. Specifically, the augmentation provides an efficient cue for the similarity information of unlabeled fundus images, assisting the supervision from the labeled data. By mining the consistent correlations from augmentation and raw images, the ACCN can discover subtle lesion features by clustering with fewer annotations. Experiments on Messidor and APTOS 2019 datasets show that the ACCN surpasses many state-of-the-art methods in a semisupervised manner.

## 1. Introduction

Diabetic retinopathy (DR) is one of the most prevalent complications caused by diabetes, which may cause intermittent or even permanent blindness [1–3]. Ophthalmologists often judge the severity of DR based on the features of the disease and the number of lesions, such as observing the characteristics of microaneurysms, hemorrhages, soft exudates, and hard exudates [4, 5]. Recognized by international authorities [6, 7], the severity of DR can be categorized into the following five levels: normal, mild, moderate, severe nonproliferative, and proliferative; these can be summarized into two main categories: normal and abnormal or nonreferable and referable symptoms [7–9]. If the retina is in the pathological state of DR for a long time, the blood vessels in the eye will eventually become blocked, eventually leading to decreased vision and even blindness. Therefore, it is essential to detect DR early and grade the DR severity in patients because early correct and timely treatment can largely avoid the deterioration of the disease.

In clinical diagnosis, DR detection mainly relies on the careful comparison of colorful fundus images by ophthalmologists. Recently, as the number of diabetic patients has increased yearly, the number of subjects to be tested has become vast, bringing a significant burden on ophthalmologists and DR experts who waste much time observing fundus images. Therefore, it is necessary to develop computer-aided diagnosing models to efficiently reduce the workload and inspection time for ophthalmologists and experts, achieving real-time DR diagnosis for patients.

To solve the automatic DR grading, early attempts [10–13] are inclined toward exploiting traditional machine learning methods on manual features, limited by specific feature extraction skills and experience. Aiming at this weakness, deep learning has become a popular solution for DR grading with many successful applications [14, 15] because it can automatically learn critical features from fundus images, supervised by accurate annotations. However, these models often depend on a large number of labeled fundus images, whose discriminant information only occurs in subtle blood vessels. The DR grading annotators must master the professional medical knowledge to support them, manually finding key features to decide on actual DR severity, which is a highly time-consuming workload. Thus, high-quality labeled data are scarce, making the supervised DR grading model hard to accomplish.

To save the expensive annotating work in real applications, this paper attempts to solve automatic DR grading in a semisupervised manner to integrate unlabeled data into the training stage because clinical inspection can produce many unlabeled fundus images containing important potential information. Thus, the most crucial task of this paper is to train a robust DR-grading model from massive unlabeled data assisted by fewer annotations, as shown in Figure 1. Extracting more identical information from unlabeled fundus images becomes a top priority, and the data consistency of unlabeled data is vital for feature learning in our work [16–19]. Inspired by previous works, we make more efforts to mine consistent correlations between raw fundus images and their augmentations, which preserve the consistent discriminative information but suffer from image transformations, such as geometric transformation, color space augmentation, random erasing, generative adversarial networks, and neural style transfer.

In this paper, we propose an augmentation-consistent clustering network (ACCN) to alleviate the laborious annotating workload in clinical application, which straightforwardly mines the consistent inner correlations among fundus image augmentations and dynamically conducts weight clustering to utilize the sufficient unlabeled data, absorbing fewer annotated fundus images. As the discriminant cues indicating DR grades are subtle in fundus images, the augmentations from raw images can help the ACCN spread the information from annotated data to unlabeled images. Besides, an online memory unit is introduced to dynamically update the clustering centroids, guaranteeing the global consistency between labeled and unlabeled fundus images in exploring critical information.

The main contributions of this article are summarized as follows:

1. We propose a brand-new, highly robust semisupervised framework (ACCN) to solve the DR grading problem, inspired by the consistent discriminative correlations between labeled and unlabeled fundus images with different augmentations.
2. We design a reasonable weight-clustering algorithm that benefits from an online memory unit to dynamically update the clustering centroids with global consistency, generating high-quality pseudolabels for unlabeled images and integrating annotated fundus images to explore discriminative information for DR grading.
3. We conducted experiments on the public data sets Messidor and APTOS 2019, and the results show that the ACCN is superior to many state-of-the-art DR grading methods.

## 2. Related Work

This section summarizes recent works on the diabetic retinopathy grading problem and introduces the successful computer-aided diagnosing applications of semisupervised learning.

### 2.1. Diabetic Retinopathy Grading

With the continuous development of deep learning, its application to retinal images has also achieved great success. Recently, some new research has been proposed [20–23]. For example, Sambyal et al. [20] proposed an aggregated residual transformation-based model for automatic multistage classification of diabetic retinopathy. Bhardwaj et al. [21] developed a hierarchical severity-level grading system to detect and classify DR ailments. Bodapati et al. [22] presented a hybrid deep neural network architecture with a gated attention mechanism for automated diagnosis of diabetic retinopathy. Math et al. [23] designed a segment-based learning approach for diabetic retinopathy detection, which mutually learns classifiers and features from the data and achieves significant development in diabetic retinopathy recognition.

However, the methods mentioned above require a large amount of labeling information. Medical labeling is well known to be expensive and time-consuming, which many institutions cannot afford. This significantly constrains the transferability of these developed DR grading systems.

### 2.2. Semisupervised Learning in Medical Image Classification

In recent years, medical imaging technology has been fully developed for clinical applications [24–26]. In medical image analysis, annotation is often difficult to obtain because it is expensive and labor-intensive. Semisupervised learning to relieve the pressure of labeling has provided great help to a certain extent. In recent years, some studies have successfully applied the semisupervised framework to medical image analysis [27–31]. Wang et al. [27] incorporated virtual adversarial training on both labeled and unlabeled data into the course of training, self-training, and consistency regularization to effectively exploit useful information from unlabeled data. Calderon et al. [28] explored the impact of using unlabeled data through the implementation of a recent approach known as MixMatch for mammogram images. Pang et al. [29] developed a radionics model based on a semisupervised GAN method to perform data augmentation in breast ultrasound images. Liu et al. [30] proposed a self-supervised mean teacher for chest X-ray classification that combines self-supervised mean-teacher pretraining with semisupervised fine-tuning. Bakalo et al. [31] designed a deep learning architecture for multiclass classification and localization of abnormalities in medical imaging illustrated through experiments on mammograms.

In this paper, we propose a novel augmentation-consistent clustering network (ACCN) for semisupervised diabetic retinopathy grading on fundus images, exploring the discriminative information learned from plentiful unlabeled data and fewer annotated fundus images.

## 3. Method

Aiming to explore the discriminant information from massive unlabeled fundus images, we design a novel semisupervised DR grading approach, the augmentation-consistent clustering network (ACCN), to assist the supervised model trained by fewer annotated data. The ACCN utilizes consistent learning and weight clustering on easily accessible unlabeled data with the help of fewer annotations to achieve the semisupervised diabetic retinopathy grading task. In detail, the ACCN first considers the category correlations among unlabeled fundus images, maintaining consistency with different augmentations. Then the trained model from annotated fundus images is utilized as the baseline network, and the ACCN deploys a clustering algorithm to weight their CNN features to calculate the pseudolabels for unlabeled images. Finally, we utilize the real annotations and pseudoannotations to train the network parameters. The whole workflow for the ACCN is illustrated in Figure 2, and the symbols are summarized in Table 1.

### 3.1. Augmentation-Consistent Learning

In semisupervised DR grading work, the most crucial task is the exploration of unlabeled retinal images. At the same time, the augmentation in deep learning is a popular and easily conducted process to produce various transformations for unlabeled raw fundus images, containing consistent identity information but close to realistic scenarios [19, 32]. Thus, the ACCN first conducts reasonable augmentations for raw retinal images to generate diverse data with the same category and then employs a convolutional neural network to learn appearance feature representations for the augmented images.

In the ACCN, we adopt augmentation anchoring technology [19, 32] that utilizes the pseudolabels that come from weakly augmented samples as the “anchor” and align the strongly augmented samples to the “anchor.” Notably, the weak augmentation *A*_weak_ in our method contains a random cropping followed by a random horizontal flip, and the strong augmentation sequence A_strong_={A_strong_^1^, A_strong_^2^, ⋯, A_strong_^k^} is achieved by RandAugment and a fixed augmentation strategy that contains a sequence of image transformations.

Because the labeled images contain sufficient grading information to find samples in the same category, with no need to generate much more augmented images, we only process the annotated retinal image *x*_*i*_^*l*^ by weak augmentation to produce an “anchor” ${\tilde{x}}_{i}^{l}$,

(1) $$\begin{array}{c} {\tilde{x}}_{i}^{l}=A_{\mathrm{weak}}\left(x_{i}^{l}\right), \end{array}$$

while the unlabeled fundus image *x*_*u*_^*l*^ should be transformed into an image sequence by strong augmentations to produce more strongly augmented samples to form sufficient training data in the same category. Thus, we utilize the strong augmentation series to generate their augmentations:

(2) $$\begin{array}{c} {\tilde{X}}_{j}^{u}={\left\{A_{\mathrm{strong}}^{k}\left(x_{j}^{u}\right)\right\}}_{k=1}^{K}, \end{array}$$

where ${\tilde{x}}^{u}$ denotes *K* strongly augmented unlabeled fundus images from *A*_*strong*_.

Through the above-mentioned augmentations, we can obtain the weak augmented annotated image ${\tilde{\text{x}}}_{\text{i}}^{l}$ and strong augmented unlabeled fundus images ${\tilde{\text{X}}}_{\text{j}}^{u}$, which are intended to supervise the model training to analyze the images from multiple angles and extract more critical features.

As for feature learning, the ACCN employs the ResNet-50 architecture [33] as the feature extractor for fundus images and their augmentations due to its excellent performance in medical imaging. Particularly, the feature extractor is defined by *G* for annotated and unlabeled retinal images, and the feature vector *G*(*·*) is transformed into a probability vector by a classifier *F*. Taking a retinal image *x* as an example, its prediction can be mathematically represented by

(3) $$\begin{array}{c} P\left(x\right)=F\left(G\left(x\right)\right). \end{array}$$

Essentially, the weak augmented images enlarge the scale of labeled data to compose a labeled set $X^{l}=\left\{x_{1}^{l},x_{2}^{l},\cdots ,x_{N_{l}}^{l}\right\}\cup \left\{{\tilde{x}}_{1}^{l},{\tilde{x}}_{2}^{l},\cdots ,{\tilde{x}}_{N_{l}}^{l}\right\}$, training the feature extractor and classifier by labeled cross-entropy (lce) loss:

(4) $$\begin{array}{c} L_{lce}=-\sum_{x_{i}\in X^{l}}y_{i}^{l}\log\;F\left(G\left(x_{i};W_{G}\right);W_{F}\right), \end{array}$$

where *W*_*G*_ and *W*_*F*_ represent the network parameters of the feature extractor and the classifier, respectively.

Similarly, the strong augmentations for unlabeled images produce the transformed samples with the same category as raw images. Thus, we also introduce an augmentation-consistent (ac) loss to enforce that the classifier predicts the consistent probability vectors for the correlated augmentation and raw fundus images:

(5) $$\begin{array}{c} L_{ac}=\sum_{x_{j}\in X^{u},{\tilde{x}}_{j}\in {\tilde{X}}_{j}^{u}}\left\|P\left(x_{j}\right)-P\left({\tilde{x}}_{j}\right)\right\|, \end{array}$$

where *X*^*u*^={*x*_1_^*u*^, *x*_2_^*u*^, ⋯, *x*_*N*_*u*__^*u*^} denotes the set of unlabeled retinal images.

Benefiting from the labeled cross-entropy loss *L*_*lce*_ and augmentation-consistent loss *L*_*ac*_, the feature extractor *G* and classifier *F* can learn a lot from the discriminative consistency between augmentations and raw images, especially from the unlabeled retinal images. Hence, the backbone network in the ACCN possesses quite an inferential capability for unknown retinal images.

### 3.2. Weight Clustering Unit

Even though the consistency information has been extracted from unlabeled images, accurate diabetic retinopathy grading cues are implied in the annotations. In recent years, pseudolabels have become an essential research topic in unlabeled image analysis [34–36]. However, simply introducing a pretrained fully connected classifier *F* by the limited labeled data does not contain robust identification ability; thus, it cannot effectively extract the internal association between the unlabeled feature representations because the augmentation consistent loss is short of the annotations. To address this weakness, the ACCN designs a weight clustering unit to mine the mutual relationships between unknown samples and their pseudolabels.

Specifically, we calculate the estimated centroid *c*_*k*_ for each class according to the primary outputs from the trained classifier *F*:

(6) $$\begin{array}{c} c_{k}=\frac{\sum_{x_{i}^{u}\in X^{u}}\delta_{k}\left(F\left(G\left(x_{i}^{u}\right)\right)\right)G\left(x_{i}^{u}\right)}{\sum_{x_{i}^{u}\in X^{u}}\delta_{k}\left(F\left(G\left(x_{i}^{u}\right)\right)\right)}, \end{array}$$

where *δ*_*k*_ corresponds to the *k*-th element output by softmax. Then, we calculate the distance between each unlabeled feature and each centroid to generate pseudolabels according to the nearest neighbor principle:

(7) $$\begin{array}{c} y_{j}^{u}=\arg\underset{k}{\min}d\left(G\left(x_{j}^{u}\right),c_{k}\right), \end{array}$$

where *d*(·, ·) denotes the Euclidean distance measure. In this way, we induce the prediction model focus on some samples around the decision boundary and explore more discriminative information by the weight clustering unit.

It should be noted that weight clustering is supported by iterative epochs to update the centroids. This means that multiple clustering is required in each batch, producing different local centroids. This may cause much more centroid deviation with wrong pseudolabeled annotations. To avoid this problem in our ACCN model, we design a dynamic centroid memory {*M*_*k*_}_*k*=1_^*N*_*c*_^ to store the temporary global centroids in each batch, where *M*_*k*_ is the *k*-th class center and *N*_*c*_ represents the number of image categories. Besides, the updated strategy for the global centroid is as follows:

(8) $$\begin{array}{c} M_{k}=\left(1-\eta_{t_{k}}\right)M_{k}+\eta_{t_{k}}c_{k}, \end{array}$$

where *η*_*t*_*k*__=*e*^−*t*_*k*_^ represents the updating rate of grade *k* and *t*_*k*_ denotes the number of categories *k* that appeared in the previous batch.

Finally, we minimize the distance between the local and global centroids in each batch by a global consistent (gc) loss:

(9) $$\begin{array}{c} L_{gc}=\frac{1}{N_{c}}\sum_{k=1}^{N_{c}}{\left\|M_{k}-c_{k}\right\|}_{2}. \end{array}$$

By advancing the above-mentioned relationship, we can alleviate the problem that wrong pseudolabeled samples cannot be correctly distinguished, which also improves the effect of diabetic retinopathy grading.

By the weight clustering unit, we can obtain reasonable pseudoannotation for the unlabeled retinal images. This supports us to conduct the annotation level supervised training from unlabeled fundus data and their strong augmentations $X^{u}=\left\{x_{1}^{u},x_{2}^{u},\cdots ,x_{N_{u}}^{u}\right\}\cup \left\{{\tilde{X}}_{1}^{u},{\tilde{X}}_{2}^{u},\cdots ,{\tilde{X}}_{N_{u}}^{u}\right\}$ corresponding to their pseudolabels {*y*_1_^*u*^, *y*_2_^*u*^, ⋯, *y*_*N*_*u*__^*u*^}, according to a pseudo-cross-entropy (pce) loss:

(10) $$\begin{array}{c} L_{pce}=-\sum_{x_{j}\in X^{u}}y_{j}^{u}\log\;F\left(G\left(x_{j};W_{G}\right);W_{F}\right). \end{array}$$

### 3.3. Final Loss for ACCN Model

As described above, our semisupervised diabetic retinopathy grading approach ACCN is composed of two crucial modules, namely, an augmentation-consistent learning and a weight clustering unit, attached with labeled cross-entropy loss *L*_lce_, augmentation-consistent loss *L*_ac_, global-consistent loss *L*_gc_, and pseudo-cross-entropy loss *L*_pce_.

To update all trainable parameters in the ACCN, we integrate the final loss into the network with balance parameters:

(11) $$\begin{array}{c} \underset{W_{G},W_{F}}{\min}L=L_{lce}+\gamma_{1}L_{ac}+\gamma_{2}L_{gc}+\gamma_{3}L_{pce}, \end{array}$$

where *γ*_1_, *γ*_2_, and *γ*_3_ are parameters to balance different loss functions.

## 4. Experiments

### 4.1. Database Description

In this section, we evaluate the proposed augmentation-consistent clustering network by training on the publicly available dataset Messidor [37]. In detail, Messidor [37] contains approximately 1200 digital fundus images obtained by using a Topcon TRC NW6 nonmydriatic camera. The sizes of fundus images are 440 *×* 960, 2240 *×* 1488, or 2304 *×* 1536 in, and ophthalmologists labeled each image. According to the DR severity, Messidor classifies the fundus images into one of the four grades, namely, normal and no lesion (*R*0), mild (*R*1), severe nonproliferative (*R*2), and proliferative (*R*3) retinal images. The data distribution of Messidor in each grade is described in Table 2, and the popular DR grading task of normal/abnormal classification is summarized in Table 3. The distribution shows that the common challenging problem is the data imbalance, which may influence the model training.

### 4.2. Experimental Settings

This paper conducts normal/abnormal DR grading experiments, dividing the dataset into 600 training images and 600 testing samples. In detail, labeled retinal images in the training data contain 400 labeled fundus images, including 200 positive cases and 200 negative images. As for the unlabeled training data, they contain 46 positive cases and 154 negative images. In addition, we chose the left 600 retinal images as testing data, which contain 300 positive and 300 negative cases. The entire experimental process is completed using the PyTorch framework under GeForce 2080TI GPU. Precisely, each retinal image is adjusted to 512 *∗* 512 pixels before inputting it to the network, and the batch size is set to 8. Besides, we use ResNet-50 as the backbone, and the classifier is composed of linear layers. For parameter settings, the learning rate is set to 0.001, and balance parameters [*λ*_1_, *λ*_2_, and *λ*_3_] are [0.6, 0.3, and 0.8, respectively] to perform the best DR grading results. In addition, the training process spends around 2.5 minutes per epoch, and the evaluation for testing images takes 5 milliseconds per fundus image.

To measure the experimental performance, we adopt the popular indicators to compare and evaluate our models: specificity (SPE), sensitivity (SEN), accuracy (ACC), and the area under the ROC curve (AUC).

### 4.3. Comparison with Other Methods

#### 4.3.1. Performance on Messidor

In order to demonstrate the performance of the ACCN on DR grading, we compare with different baseline methods for the normal/abnormal DR grading task. As to the compared methods, we choose the manual grading results from two experts [38] and introduce two experimental methods used in [39], which emphasize the role of multiple filter sizes in learning fine-grained discriminant features and proposes two deep convolutional neural networks, combining kernels with a multiple loss network and a V_gg_ network. The normal/abnormal fundus image classification results on Messidor are reported in Table 4, and our ACCN framework achieves the highest accuracy of 89.8%, sensitivity of 93.0%, specificity of 86.7%, and AUC of 93.6%, outperforming the supervised DR grading model and experts. What needs to be emphasized is that our ACCN model only utilizes 400 annotated retinal images and other training data is unlabeled while the compared models require fully annotated retinal images and experts require long-term professional training. Therefore, the excellent performance of our ACCN in a semisupervised manner proves that it can save us from depending on expensive annotating networks in significant applications for DR grading.

Besides, we choose two existing semisupervised medical image classification methods [30, 41] to compare with our ACCN model. S^2^MTS^2^ [30] combines self-supervised mean-teacher pretraining with a semisupervised fine-tuning method to solve the multilabel chest X-ray classification; SRC-MT [41] proposes a sample relation data consistency paradigm to effectively extract unlabeled data by modeling the relationship information among different medical image samples. To compare the ACCN with them, we implement their public available code on the Messidor dataset with the same settings. The results are summarized in Table 4, proving that our ACCN approach is superior to those semisupervised medical image classification methods, with considerable improvements in each metric. Although our method outperforms some supervised methods, there is still a gap with advanced supervised methods, and the ACCN still has the potential to be explored to reach the supervised performance.

### 4.4. Visual Analysis for ACCN

This article outlines two popular visualizations for the ACCN to make it generally available for the diabetic retinopathy grading task. First, the ROC curve is shown in Figure 3, and our approach achieves an AUC of 0.96 on the Messidor dataset. Besides, we utilize 600 testing fundus images and illustrate the classification results in the confusion matrix (Figure 4). The confusion matrix can quickly visualize the proportion of various misclassified categories into other classes. From the results, the ACCN model correctly classifies the 279 abnormal and 261 normal fundus images, with 89.9% accuracy. Summarizing the above-mentioned visualization results, we can see that our ACCN model effectively utilizes a large amount of unlabeled data with fewer annotations to solve the semisupervised DR grading task well.

At the same time, we calculate the loss reduction during model training, illustrated in Figure 5. The overall loss reveals a downward trend, and the regeneration of pseudolabels causes the ups and downs in the first half by clustering within the batch. After adding the global-consistent loss, the clustering centroids are dynamically updated more reasonably, with stable loss convergence. This demonstrates that our ACCN can rapidly train a semisupervised DR grading model and the global-consistent loss significantly improves the convergence.

### 4.5. Performance on Other DR Grading Datasets

This article also chooses another publicly available DR grading dataset, APTOS 2019, in the normal/abnormal DR experiments to provide the transferability of the proposed ACCN approach. APTOS 2019 [42] was proposed in the APTOS 2019 diabetic retinopathy classification contest, which was organized by the Asia Pacific Tele-Ophthalmology Society. It comprises 3662 retinal images from fundus photography with available annotations captured from multiclinics with different imaging conditions at Aravind Eye Hospital in India. Concretely, this dataset contains five classes for training the ACCN, and the data are highly imbalanced, as summarized in Table 5. Compared to Messidor, APTOS 2019 is more challenging because it contains five grades on DR and it can prove the effectiveness of our ACCN model more sufficiently on normal and abnormal DR classification, and the detailed division of different DR grades can be found in Table 4.

From Table 6, it can be found that the ACCN has reached a high accuracy of 93.4%, sensitivity of 91.0%, specificity of 95.7, and AUC of 0.984. These results mean that the ACCN can effectively extract the internal connections among unlabeled retinal images in different datasets and it can successfully solve the DR grading problem with fewer annotations when transferred to other application scenarios.

## 5. Further Analysis

This section further discusses the impacts of major components and parameters on the ACCN approach to the semisupervised DR grading task, including the labeled data, augmentation-consistent learning, and the weight clustering unit.

### 5.1. The Impact of Labeled Fundus Images

This paper attempts to solve the DR-grading task with fewer annotations. Thus there are very few high-quality samples with accurate labels for DR diagnosis. To measure the impacts of labeled data, we use accuracy to test how the number of labeled retinal images influences the ACCN performance on the Messidor dataset. From the results in Figure 6, it can be observed that the DR grading accuracy rapidly increases from 68.7% to 75.2% as the number of labeled fundus images increases from 50 to 100 and it mildly increases from 75.2% to 89.8% when the number of labeled data is between 100 and 400. Finally, the ACCN model achieves an accuracy of 93.4% when it is fully supervised.

The above-mentioned experimental results show that the proposed semisupervised model can work well using a relatively small number of labeled samples, with fewer annotating costs than existing supervised DR grading models. However, using the proposed ACCN approach still requires a certain amount of labeled samples to obtain a higher classification accuracy. A similar trend and conclusion can also be observed from sensitivity, specificity, and AUC.

### 5.2. The Impact of Augmentation-Consistent Learning

The first dominating method in the ACCN is the augmentation-consistent learning module, which generates weak and strong augmentations for annotated and unlabeled training images, respectively, and conducts consistent feature learning for the raw images and their augmentations. To weigh the impact of this module, we only employ raw images to conduct the weight clustering network and assign pseudolabels. The results are reported in Table 7 (ACL). Concretely, the ACL module improves the DR grading performance with an accuracy of +13.5%, sensitivity of +14.7%, specificity of +12.4%, and AUC of +14.6%. This further certifies that the novelties of our proposed augmentation-consistent learning mechanism are beneficial to the semisupervised DR grading task.

### 5.3. The Impact of Weight Clustering

We then analyze the influence of the weight clustering module. We remove the entire clustering module and directly use the prediction vector of the high-confidence sample after the softmax output as the pseudolabel for training. The effect of normal/abnormal DR classification on the Messidor dataset is that the accuracy has dropped by 8.1%, which demonstrates that the ACCN employing a weight clustering unit to explore the internal relationship between unknown samples is effective in semisupervised DR grading task. Compared to the supervised models in the study by Holly et al. [39], our model achieves a competitive AUC of 86.2% when removing the WLU. It benefits from the proposed augmentation-consistent learning module and further proves the effectiveness of our semisupervised learning approach.

### 5.4. The Impact of Positive Cases in Unlabeled Data

The positive proportion of unlabeled data is an important factor affecting the final performance for the semisupervised diabetic retinopathy grading problem. We finally discuss the influence of the positive proportion of unlabeled training data by changing the proportion of positive cases in unlabeled data. The results on the Messidor dataset are summarized in Figure 7, revealing that the accuracy of performance decreases with increasing positive proportion in unlabeled training. This demonstrates that the positive cases in labeled training data provide more discriminative information than the ones in unlabeled data. Thus, the balanced distribution of negative and positive cases both in labeled and unlabeled data is important for the semisupervised diabetic retinopathy grading task. In addition, under the premise that the number of labeled samples remains unchanged, we record experimental results employing different proportions of positive samples (unlabeled). The result is shown in Figure 8.

## 6. Discussion and Conclusion

For the real application of diabetic retinopathy grading, the lack of labeled data is the main challenge that limits the application of deep learning. This is probably due to the following reasons. First, the lesion indicating DR is always subtle in digital fundus images, so labeling retinal images require expertise in long-term training, and hiring experts to annotate is very expensive and time-consuming. Second, medical data, especially images for human diseases, become difficult to collect due to rigorous privacy issues. Finally, the diseases that require the aid of computer vision are often complex, and the model training must use sufficient data, making the fundus image annotation more complicated.

To address the above-mentioned challenges, we propose an augmentation-consistent clustering network (ACCN) approach for semisupervised diabetic retinopathy grading, which can mine internal correlations among unknown samples assisted by fewer annotations. The proposed model can compensate for the lack of labeled data in the following ways. (1) The augmentation-consistent learning generates weak and strong augmentations for annotated and unlabeled fundus images and provides inherent consistent information by labeled cross-entropy and augmentation-consistent losses. (2) A weight clustering unit is designed to calculate the pseudolabels for unknown retinal images with a dynamically clustering algorithm, which utilizes weight centroids to cluster in a global-consistent manner. (3) The DR classification model is further trained by combining annotated and pseudolabeled retinal images to achieve the semisupervised diabetic retinopathy grading task. Adequate experiments on the Messidor dataset prove that the ACCN can perform effective DR classification with limited labeled data, and the extensive experiments on APTOS 2019 demonstrate the scalability of our ACCN network to different domains.

In future, we will work on the unsupervised learning approach to conduct fundus image classification without any annotations. Besides, we will focus on diabetic retinopathy grading in multiple stages to provide a more accurate diagnosis for ophthalmologists.

## Figures and Tables

**Figure 1:** Analysis diagram of our semisupervised DR-grading solution.

**Figure 2:** Scheme of the augmentation-consistent clustering network. First, different augmentations for annotated and unlabeled fundus images are generated in a weak and a strong manner, respectively, and consistent feature learning is conducted to train a robust feature extractor. Then, the unlabeled feature representations are fed into a weight-clustering unit to assign pseudolabels with dynamically updating memory in model training. Finally, the pseudolabels and corresponding unlabeled retinal images are utilized to optimize the whole network for solving the DR grading task with fewer annotations.

**Figure 3:** ROC curve of the proposed ACCN model for normal/abnormal DR grading on the Messidor dataset.

**Figure 4:** Normal/abnormal DR classification on the Messidor dataset.

**Figure 5:** Loss curve of the ACCN for model training on the Messidor dataset.

**Figure 6:** DR classification performance with different numbers of labeled data.

**Figure 7:** The accuracy results of different positive proportions in unlabeled training data.

**Figure 8:** The accuracy results with different ratios of positive samples in unlabeled data.

**Table 1:** The symbol summary.

Symbol	Meaning
*x*_*i*_^*l*^	The *i*-th annotated retinal image
*x*_*j*_^*u*^	The *j*-th unlabeled retinal image
*A*_weak_	The weak augmentation
A_strong_	The collection of strong augmentations
${\tilde{x}}_{i}^{l}$	The weak augmented image for *x*_*i*_^*l*^
${\tilde{X}}_{j}^{u}$	The collection of strong augmentations for *x*_*j*_^*u*^
*G*	The feature extractor
*F*	The classifier
*X* ^*l*^	The labeled raw images and their augmentations
*X* ^*u*^	The set of unlabeled raw images
*X*_*u*_	The unlabeled raw images and their augmentations
*c*_*k*_	The local centroid for *k*-th class
*y*_*j*_^*u*^	The generated pseudolabel
*M* ^*k*^	The global centroid

**Table 2:** The class distribution of datasets.

Label	Messidor
DR 0	546
DR 1	153
DR 2	247
DR 3	254

**Table 3:** The popular classification task on DR grades.

Label	Description
DR grading	DR 0/DR 1/DR 2/DR 3
Normal/abnormal DR	DR 0/DR 1, DR 2, DR 3

**Table 4:** Compared performance on Messidor.

Methods	Accuracy	Sensitivity	Specificity	AUC
Expert A [38]	87.8	—	—	92.2
Expert B [38]	76.4	—	—	86.5
Holly et al. [39]	87.1	88.2	85.7	87.0
Holly et al. [39]	85.8	91.6	80.3	86.2
Odena et al. [40]	94.7	95.4	95.1	96.7
S^2^MTS^2^ [30]	86.7	88.7	84.8	86.3
SRC-MT [41]	85.8	86.4	85.2	84.8
ACCN	89.8	93.0	86.7	96.0

**Table 5:** The class distribution of APTOS 2019.

Label	APTOS	Division
DR 0	1805	Normal
DR 1	370	Abnormal
DR 2	999	Abnormal
DR 3	193	Abnormal
DR 4	295	Abnormal

**Table 6:** Experimental results on APTOS 2019.

Methods	Accuracy	Sensitivity	Specificity	AUC
ACCN	93.4	91.0	95.7	98.4

**Table 7:** The contributions of the major steps in ACCN (%).

Target	Accuracy	Sensitivity	Specificity	AUC
ACL	+13.5	+14.7	+12.4	+14.6
WLU	+8.1	+9.3	+7	+9.8

## Data Availability

The datasets used and/or analyzed during the present study are available from the corresponding author on reasonable request.
